The article "Assessing wellbeing: Profiling and socioeconomic status of Kenyir Lake side community, Malaysia" was published in 2023. Journal: Heliyon.

# Assessing wellbeing: Profiling and socioeconomic status of Kenyir Lake side community, Malaysia

**DOI:** 10.1016/j.heliyon.2023.e16399

**Published:** 2023-05-28

**Authors:** Norhayati Ab Manaf, Nor Hayati Sa’at, Nurul Aisyah Awanis A Rahim, Siti Nor Adawiyah Azzahra Kamaruddin, Siti Salina Abdullah, Khatijah Omar

**Affiliations:** a Institute of Tropical Biodiversity and Sustainable Development, University Malaysia Terengganu, Terengganu, Malaysia; b Faculty of Business, Economics and Social Development, University Malaysia Terengganu, Terengganu, Malaysia; c Faculty of Business Management, University Sultan Zainal Abidin, Terengganu, Malaysia

**Keywords:** Development, Rural community, Kenyir lake, Well-being

## Abstract

The Kenyir Lake side community offers numerous advantages to the local community. However, the problems of backwardness and poverty have been identified as the government's main challenges in its efforts to develop the community and maximise the advantages. Therefore, this study was conducted to identify the Kenyir Lake community's profile and assess its well-being. The study was conducted in three sub-districts near Tasik Kenyir, namely Kuala Berang, Hulu Telemong, and Jenagor, with a total of 510 respondents, who are heads of households (HOH). This study was carried out using a quantitative approach using questionnaire with a simple random sampling method. The findings of this study offered demographic profiling and discovered nine indicators of well-being, namely 1) Life Achievement, 2) Health Level, 3) Family Relationship, 4) Community Relationship, 5) Spiritual Level, 6) Safety Level and Social Problems, 7) Income or Finance, 8) Basic Facilities, and 9) Communication Technology. The study found that most respondents are satisfied with their lives now compared to 10 years ago. This study will help many parties to develop the Kenyir Lake Side Community, starting from the local authorities to the highest administration in the country.

## 1 Introduction

Nowadays, the main challenge in a societal development is to improve the standards of living in line with rising living costs. The government has provided various development needs that can be enjoyed by all groups to face the challenges of the Industrial Revolution 4.0 (IR4.0). Indeed, the government is working hard to improve the socio-economic status by planning and providing various development needs that can be enjoyed by all groups in Malaysia [44]. The progress and development are highly dependent on the community members who are striving to achieve its well-being. The involvement and commitment of all community members are vital in developing values of unity to plan, manage, and implement shared needs to achieve the well-being of their lives [2]. A community's capacity is built when its members participate actively in development programmes [24]. It is a country's greatest challenge to improve its performance in education, health, housing, and employment [39].

The article "Assessing wellbeing: Profiling and socioeconomic status of Kenyir Lake side community, Malaysia" was published in 2023. Journal: Heliyon.

Social well-being is highly dependent on the quality of life achieved by a group of communities, including rural communities [22]. The problem of rural communities' well-being is universal. Backwardness and poverty have been identified as significant challenges faced by the government to develop communities effectively. Most developed countries face similar issues in the development process and well-being of their populations, especially the rural communities. Rural communities, especially the lakeside communities of Kenyir Lake, are still unable to compete. In fact, they are still victims of the prejudice of outside capitalists who invest in their place. Thus, the local community is only seen as passengers with no direction or mere observers. Hence, they are often considered only qualified as unskilled labour contributors who cannot take advantage of the opportunities created by the ongoing development in their community [34].

The local community's willingness to participate in a development programme is a crucial factor contributing to the success of development activities or programmes implemented. However, research proves that various factors frequently hamper local communities' willingness to participate in development programmes. The development of Kenyir Lake as the best tourist destination is one of the tourism development programmes implemented rapidly in Terengganu. Making Bayas Island in Kenyir Lake the first ‘island in a lake’ in Asia to be declared a duty-free zone is one of the main attractions. Therefore, this study aims to identify the Kenyir Lake community's profile and assess its well-being. The specific objectives of this study, which are to identify the demographic profile of the community nearest to Kenyir Lake, identify their socioeconomic status, and analyse the well-being of the community based on the development at Kenyir Lake.

## 2 Literature review

### 2.1 The development of Kenyir Lake

Economically, the community in Hulu Terengganu can obtain various benefits from Kenyir Lake, including the new sector employment opportunities there, which is a source of unique attractions in terms of the environment, geological characteristics, and rich natural resources. This privilege creates the local community with various employment and workforce opportunities. Among them are tourism, agriculture, services, hospitality, homestays, and aquaculture [43]. Now, the establishment of various infrastructure and latest attractions has created various new job opportunities at Kenyir Lake, such as boat drivers, tour guides, travel agency employees, hotels and chalets, retailers, restaurants, middlemen (wholesalers), gardeners, farmers, freshwater fish farmers, security officers, interpreters and translators, and cottage industry entrepreneurs as well as indigenous product entrepreneurs.

The article "Assessing wellbeing: Profiling and socioeconomic status of Kenyir Lake side community, Malaysia" was published in 2023. Journal: Heliyon.

According to KETENGAH Annual Report (2018) [18], which stated the information from the World Tourism Organization (UNWTO), from 2013 to 2017, global international tourist arrivals recorded an increase of 21.6% from 1087 million tourist arrivals in 2013 to 1322 million in 2017. Tourism is the second largest source of foreign exchange inflows in Malaysia. The tourism industry also contributed 14.8% of the country's GDP, or RM182.4 billion, in 2016, up 9.4% from the previous year.

Table 1 shows that the number of tourists visiting Kenyir Lake increases each year. Every year, this report of tourist arrivals has boosted the socio-economic development of the locals. The recognition of Geopark Kenyir at the national and international levels will create more job opportunities, given the annual increase in the number of tourists. To increase the added value to the rural economy, KETENGAH has developed a conducive business environment to provide room for economic and entrepreneurial activities, indirectly providing job opportunities for the locals. KETENGAH conducted four projects through an allocation of RM6,797,939.00 with an expenditure performance of RM6,438,973.00 (94.72%). A total of 20 units of retail space and 28 units of workshops have been provided. It is expected to establish business opportunities to 60 entrepreneurs and provide job opportunities to 177 employees [18].

**Table 1:** Number of tourist entries in lake kenyir from 2006 to 2017.

Year	No.
2006	60,532
2007	92,199
2008	133,569
2009	189,388
2010	225,570
2011	275,241
2012	397,005
2013	467,678
2017	808,336

Source [17]:

These job opportunities will also be formed through several other projects, such as Kenyir Lake Resort and Houseboat on Lake Kenyir (geo-tourism). In line with this plan, the workforce must carry out hotel operations and golf course landscape management, such as reception, food and beverage (F&B), caddy and housekeeping, and tourism and homestay industry services.

In addition, the employment growth in the tourism, services, and hospitality sectors impacts the local socio-economic environment and will improve the population's communication skills. Mechanization, technology, and agricultural inputs have all been part of the agriculture and aquaculture sector's modernization strategy. Aquaculture and caged livestock have begun to grow in Kenyir Lake due to market demand for caged fish products. The capacity of the Kenyir Lake area's rivers has been utilised. Meanwhile, the tourism sector has natural assets, such as waterfalls, rivers, and forests that have not been fully utilised by various parties in services. The diversity of natural heritage at Lake Kenyir indirectly contributes to increasing tourist arrivals, expanding the market for rural industrial enterprises' support services and products.

The article "Assessing wellbeing: Profiling and socioeconomic status of Kenyir Lake side community, Malaysia" was published in 2023. Journal: Heliyon.

### 2.2 Ecotourism and sustainable development

To create the ecosystem-related plans, basic training and education in heritage and environmental conservation are needed to meet the needs of workforce demand in the tourism sector to ensure sustainable development in Kenyir Lake. Heritage conservation courses are essential activities for entrepreneurs, employees, and local communities. They increase their understanding and awareness of heritage conservation challenges, such as reforestation activities, the environmental pollution impact and conservation measures, and environmental awareness campaigns. This education system is needed for hotels, resorts, chalets, and homestay operators. Indeed, this organization will provide employment opportunities to the local community, such as tour guides, who will be the most critical people in educating tourists on the privileges and diversity of heritage resources in the Kenyir area in the future. They will also serve as travel agents, introducing different geopark-based tourism products. Indirectly, tourists will learn and experience the true uniqueness of being in Kenyir.

Kenyir Lake, which is rich in natural resources, is seen as an opportunity by the state government. The state government has identified several specific sectors for economic growth, including small and medium businesses, tourism, and agriculture. This is in line with the state government's plan under the Terengganu State Economic Planning Unit (UPEN) to make Kenyir Lake an international standard ecotourism destination [12]. Ecotourism has been widely recognized as a form of nature tourism expected to contribute to conservation and development [33]. According to a series of workshops on the Terengganu State Development Direction (HPNT) 2009–2013, the State Government intends to make Kenyir Lake the focus for standard international tourism. Among the flagship projects that have been planned include making Lake Kenyir a duty-free area, Kenyir Island Hopping (KIH), and a water theme park.

Furthermore, the potential of Kenyir Lake to be developed as an ecotourism industry is a significant step towards achieving a sustainable development. KETENGAH has taken the initiative to exploit these elements of flora and fauna effectively and deeply to be interpreted into elements of tourism, such as ecological tourism, history and heritage, homestays, and adventure. Good infrastructure facilities are also developed aggressively and impressively, such as roads, water and electricity supply, communications, accommodation, landscaping, and basic amenities for the comfort of visitors [18].

The article "Assessing wellbeing: Profiling and socioeconomic status of Kenyir Lake side community, Malaysia" was published in 2023. Journal: Heliyon.

According to Ref. [5]; developing ecotourism in rural areas will assist the preservation of a viable rural society while also meeting the needs of new tourists from both within and outside the country. The local community needs to be involved to succeed in the sustainable development of ecotourism. This is in line with the recommendations by Ref. [35]; to ensure ecotourism is sustainable, the awareness and commitment of the local community around Kenyir Lake are very important. Therefore, efforts to provide awareness to entrepreneurs, employees, and local communities on heritage and environmental conservation must be implemented periodically.

The ecotourism sector in Kenyir Lake can provide various employment opportunities to the local community. This effort will only succeed if there is a direct involvement of the local community in these ecotourism-related activities. Therefore, the educational process on the sustainable development of the Kenyir Lake ecosystem needs to be carried out by the communities involved to create togetherness to preserve and conserve this local heritage.

According to Ref. [40]; community involvement is a form of individual voluntary effort by taking opportunities and shouldering societal responsibilities. Communities must go through a process of collaborating with those who can assist with their planning, management, and evaluation of their actions while also enhancing their development and well-being (Kalsom & Nor Ashikin, 2009). Along with the concept of sustainable development, quality of life is also seen from both aspects of economic balance and environmental care [3]. has explained that quality of life involves changes in society and the social system starting from the awareness of individuals to practice a healthy lifestyle and is able to meet their survival needs and free to develop the potential of the individual. Every individual who shares the same goals and viewpoints will form a community that cooperates and shows respect towards each other in the same environment [13]. To achieve sustainable development, sustainable communities must be formed based on the principles of sustainability, namely the balance between the economy, social, and environment.

The article "Assessing wellbeing: Profiling and socioeconomic status of Kenyir Lake side community, Malaysia" was published in 2023. Journal: Heliyon.

### 2.3 Community well-being

The concept of wellbeing is a dynamic process. People value it when they can demonstrate how their lives have changed for the better or worse, depending on their status. Ref. [23]. Although there are many other dimensions to the idea of well-being, income levels frequently influence it. To identify the genuine level of wellbeing, metrics based on income determination will have questionable accuracy [46]. According to Ref. [23]; the concept of well-being is wide and encompasses a variety of dimensions of life, including social, psychological, and economic ones. According to Ref. [26]; there are two types of well-being: subjective and objective. While the subjective category is measured by the level of life satisfaction attained by the individual, such as happiness and thankfulness throughout life, the objective category refers to a person's basic necessities and can be observed externally through factors like money, education, health, and housing. The maximum level of satisfaction and well-being is therefore found in subjective well-being, which is also utilised as a measure of human well-being more accurately. Social well-being is a goal for individuals, families, and communities to achieve. It is a key element that determines the core development of a community [1]. Well-being refers to a standard and quality of life that meets an individual's socioeconomic, physical, and psychological needs. Well-being is crucial to increase productivity and social mobility and strengthen social cohesion and national unity. Quality of life is one indicator to measure a society's well-being. If quality standards are achieved in education, economy, social status, moral values, and religion, it can be said that a society is in prosper [27].

According to the Malaysian Family Well-Being Index, family well-being refers to the state of the family being safe, harmonious, and satisfactory. It covers various aspects, namely spiritual, economic and financial, mental, psychosocial, health, political, and sustainability [25]. The study found six factors of well-being, namely income, education, property/asset ownership, job opportunities/increased income, job opportunities for children, and community involvement. According to Ref. [7]; all social issues, such as lack of education, health, and lack of employment opportunities are among the issues often associated with this group of people.

Several theoretical approaches can be used to apply this research on development and well-being, including the Wellbeing Theory and Maslow's Hierarchy of Needs Theory. The Wellbeing Theory includes Classical utilitarian, Neoclassical welfare theory, and New contraction approach. Based on this theory, the level of well-being can be related to the level of satisfaction and the level of pleasure that can be achieved in a person's life [32]. explained that the well-being theory is a form of social intervention that can improve human well-being. It also involves a process to control and improve the quality of life. It is also supported by Ref. [38] who states that improving well-being is parallel with the need through the provision of assistance to a person or a group of people to achieve a satisfactory standard of living and health. This shows that the study of the achievements of programs implemented by related agencies is very important to see the level of well-being of the community itself. Then, Maslow's Hierarchy of Needs Theory is also adapted to indicators of well-being and factors that are expected to have an impact on an individual's participation and readiness for implementation of the program. All the indicators and factors in Abraham Maslow's theory are considered in this study which cover i) physiological needs, ii) security, iii) love, iv) self-esteem, and v) the need for self-perfection. Maslow's theory is considered suitable for human life based on studies that have been done. Maslow's theory is suitable to be applied to measure the level of satisfaction in life and motivate people to keep moving forward. Maslow's theory is also used in various aspects, such as education, employment, administration, and counselling. This is because Maslow's Theory is a motivational theory to motivate people to progress. Therefore, various agencies, schools, and institutions have conducted research by applying Maslow's Theory in their respective sectors [4,8,21,31,41]. Based on the literature review and the theories discussed in this study, the following conceptual framework is proposed (see Fig. 1).

The article "Assessing wellbeing: Profiling and socioeconomic status of Kenyir Lake side community, Malaysia" was published in 2023. Journal: Heliyon.

**Fig. 1:** Conceptual framework of well-being.

## 3 Methodology

### 3.1 Sample and data source

The population of the study used a database from Hulu Terengganu District Office, which is responsible for the villagers in Hulu Terengganu. There are 9 districts in Hulu Terengganu, which are Hulu Berang, Hulu Telemong, Hulu Terengganu, Jenagor, Kuala Berang, Kuala Telemung, Penghulu Diman, Tanggul, and Tersat. The study took a population of Kenyir Lake Side Community in Hulu Terengganu, Malaysia. Sampling targets were the Heads of Household in three districts near Kenyir Lake. The sample of this study focused on the villages that were relocated from before the dam was built and the village near to the Kenyir Lake ecosystem. A total of three districts, namely Hulu Telemong, Jenagor, and Kuala Berang, were taken and ten villages were involved, which are Kampung Basung, Pasir Dula, Jeneris, Padang Setebu, Jenagor, Kuala Pueh, Dura, Gaung, Butut, and Telaga (see Fig. 2). To determine the sample size in this study, the researcher used the Sample Size Determination by Krejcie and Morgan Table (1970). The total of the population is 5000 people for ten villages, so the best number is 357 respondents. However, the number of respondents has increased to 510 to increase data accuracy and reduce errors during the data analysis process (See Table 2). Data collection was done for five months, from December 2018 to April 2019 and have been approved accordingly and in compliance with ethical standard by University Malaysia Terengganu which act as the founding Institution for this study. The research study entitled “Empowerment Sustainable Development of The Community Through Tasik Kenyir Ecosystem” was reviewed by the ethical committee of the Institute of Tropical Biodiversity and Sustainable Development, Universiti Malaysia Terengganu. The full name of the ethical committee is provided, which is Prof. Dr. Khatijah Binti Omar. Furthermore, the statement confirms that the study was approved to be conducted in the designated study area. The statement also confirms that the survey and informed consent provided for the research were carefully reviewed, and the study was approved by the ethics committee. Data analysis of 510 questionnaires was done by SPSS software 20. Each section and item in the questionnaire were designed to identify the dependence of Kenyir Lake side communities on the ecosystem, which also faced new development and changes due to the first duty-free zone area in Terengganu, as well as examined the aspects of socio-cultural and socio-economic changes of the community, especially around the village nearest to the Kenyir Lake ecosystem.

**Fig. 2:** Map of study area.

**Table 2:** List of respondents based on districts and villages in the study area.

Districts	Village	No. Of Respondents	Percent
Kuala Berang	Gaung	45	8.8
	Telaga	54	10.6
	Butut	48	9.4
Hulu Telemong	Basung	99	19.4
	Pasir Dula	51	10
	Padang Setebu	16	3.1
	Kuala Jeneris	27	5.3
Jenagor	Kuala Pueh	52	10.2
	Dura	83	16.3
	Jenagor	35	6.9
Total		510	100%

List of the districts and villages in the study area is stated in Table 2.

### 3.2 Variable definitions

The questionnaire was divided into two sections: the first section contained items related to the respondent's demographic information (e.g., age, resident status, and education level) and socioeconomic information (e.g., job and income). The second section involved the questions related to quality of life (See Table 3). The questions were constructed using a 5-point Likert scale. Both sections collected the descriptive data. The second section analyzed nine (9) indicators, which are 1) Life Achievement, 2) Health Level, 3) Family Relationship, 4) Community Relationship, 5) Spiritual Level, 6) Safety Level and Social Problems, 7) Income/Finance, 8) Basic Facilities, and 9) Communication Technology. The list of questions based on indicators are stated in Table 3.

The article "Assessing wellbeing: Profiling and socioeconomic status of Kenyir Lake side community, Malaysia" was published in 2023. Journal: Heliyon.

**Table 3:** Definitions of indicator and list of questions.

Indicator	Definitions	Questions
Life Achievement	An individual's perception of what he/she wants in life [45].	Q1: Satisfied with current life than before. Q3: Satisfied with achievement in life than before?
Health Level	Health is more than just the absence of disease or disability; it is a condition of whole physical, mental, and social well-being. This term has a crucial implication: mental health encompasses more than just the absence of mental diseases or disabilities. A person is in a mentally healthy state when they are aware of their own skills, able to handle life's usual stressors, able to work efficiently, and able to give back to their community. The ability of both individuals and society as a whole to think, feel, interact socially, work, and enjoy life depends on mental health. As a result, individuals, communities, and cultures all over the world should be deeply concerned with the promotion, protection, and restoration of mental health.[42].	Q2: Satisfied with current health than before. Q19: Satisfied with family health care. Q26: Satisfied with family's 3 R practices.
Family Relationship	There are three (3) theoretical perspectives, which are Functionalism, Conflict, and Symbolic interactionism. Functionalism: The family performs several essential functions for the society. It socialises children, provides emotional and practical support for its members, helps regulate sexual activity and sexual reproduction, and provides its members with a social identity. In addition, sudden or far-reaching changes in the family's structure or processes threaten its stability and weaken society. Conflict: The family contributes to social inequality by reinforcing economic inequality and by reinforcing patriarchy. The family can also be a source of conflict, including physical violence and emotional cruelty, for its own members. Symbolic interactionism: The interaction of family members and intimate couples involves shared understandings of their situations. Wives and husbands have different styles of communication, and social class affects the expectations that spouses have of their marriages and of each other [19].	Q8: Satisfied about recreation with family than before. Q11: Satisfied with current life with family than before. Q12: Satisfied with current engagement with children. Q13: Satisfied about quality time with family. Q14: Balance the work and family? Q15: Satisfied about relationship with partner. Q16: Family members play their respective roles. Q17: Satisfied with family's problem-solving.
Community Relationship	Community is frequently conceptualised as an entity that is more than the sum of its parts and, as a social grouping, captures aspects of life as they are lived and experienced together [36,37]. Community is still understood largely through these two major types, geographical and functional, and sharing the characteristics of people engaged in face-to-face communication, exchange, and interaction [10].	Q4: Satisfied with current personal relationships with others than before. Q5: Satisfied living as a member of this community than before.
Spiritual Level	The Spiritual Well-Being Scale (SWBS) measures an individual's well-being and overall life satisfaction on two dimensions: (1) religious well-being, and (2) existential well-being. Items related to religious well-being contain the word “God” and measure the degree to which one perceives and reports the well-being of his or her spiritual life in relation to God. Items related to existential well-being contain general statements that ask about life direction and satisfaction and measure the degree to which one perceives and reports how well he or she is adjusted to self, community, and surroundings [9]. Psycho-spiritual well-being is a subjective experience that incorporates both emotional health and meaning-in-life concerns. Psycho-spiritual well-being, in a positive sense, includes the following attributes: self-awareness, coping, and adjusting effectively with stress, having satisfying relationships and connectedness with others, sense of faith, sense of empowerment and confidence, and living with meaning and hope [20].	Q6: Satisfied with current religious practice than before. Q21: Satisfied with the role of religion in life. Q22: Satisfied with family's spiritual level.
Safety Level and Social Problems	Societal safety has interfaces with other safety-related areas, such as national security, sustainable development, human security, and incident management (handling of isolated accidents, common illness and ordinary criminal acts) [28].	Q9: Satisfied with current social problems in this place than before. Q10: Satisfied with current safety in this community than before. Q20: Satisfied with family safety level. Q24: Satisfied with level of pollution in this place.
Income/Finance	Income is an important proxy for measuring a person's socioeconomic status or standard of living. Household income refers to whether monetary or in-kind, that are obtained repeatedly and accrued (certainly received) either weekly, monthly, or annually, can be used to meet current needs. Household income is obtained from four main sources of income, which are income from employment whether salaried or self-employed, income from property and investments owned and income from current transfers [14].	Q7: Satisfied with current monthly financial position than before. Q18: Satisfied with family financial management.
Basic Facilities	Basic facilities are economic facilities, water and electricity supply facilities, telecommunication facilities, health services, education, public transport and communication systems, recreational facilities, workshops, and other facilities. In addition, the accessibility component of the population with the facilities provided and the extent to which the population's access to infrastructure and social facilities can improve the quality of life of the community [6].	Q23: Satisfied with basic amenities in home.
Communication Technology	Communications technology, also known as information technology, refers to all equipment and programs that are used to process and communicate information. Professionals in the communication technology field specialise in the development, installation, and service of these hardware and software systems [16].	Q25: Satisfied with family engagement in terms of communication management. Q27: Satisfied with family engagement in communication technology.

A pilot test was conducted to 30 Heads of Household on December 1, 2018 to three villages, which are Tengkawang, Kepah, and Kuala Ping, to ensure that the set of questionnaires was convenient and accurate to use to the respondents. Firstly, researchers discussed with the key informants (Heads of Village) to get a list of respondents as well as an overview and situation of the village to distribute the questionnaire.

The article "Assessing wellbeing: Profiling and socioeconomic status of Kenyir Lake side community, Malaysia" was published in 2023. Journal: Heliyon.

## 4 Results

### 4.1 Descriptive analysis (frequency and percentage) of respondent demographic information

Table 4 shows the demographic profiling of Kenyir Lake residents, consisting of communities in Kuala Berang, Hulu Telemong, and Jenagor districts. The distribution of respondents is 37.5%, 37.8%, and 24.7%, respectively, for District Kuala Berang, Hulu Telemong, and Jenagor. The total number of respondents is 510 people.

**Table 4:** Districts involved.

Districts	No.	%
**Kuala Berang**	191	37.5
**Hulu Telemong**	193	37.8
**Jenagor**	126	24.7
Total	**510**	**100.0**

Table 5 shows the distribution of respondents based on gender, age, and marital status. A total of 77.6% of respondents were male, and 22.4% were female. From the total respondents, 77.3% were married, and the rest were single, widows, and divorcees. A total of 19.8% of respondents have an age category under 40 years. The highest distribution age category was 41–60, with 48.6%. Meanwhile, the age category over 60 years is 31.5%.

**Table 5:** Gender, age, and marital status categories.

Gender	No.	%
**Male**	396	77.6
**Female**	114	22.4
**Total**	510	100.0
Age	**No.**	**%**
**35 years and below**	54	10.6
**36 until 40 years**	47	9.2
**41 until 50 years**	101	19.8
**51 until 60 years**	147	28.8
**61 until 65 years**	67	13.1
**65 years and above**	94	18.4
**Total**	510	100.0
Marital status	**No.**	**%**
**Single**	39	7.6
**Married**	394	77.3
**Widows**	67	13.1
**Divorcees**	10	2.0
**Total**	510	100.0

Next, Table 6 shows the respondents' resident's status and duration of stay. A total of 66.9% are the original residents of Kenyir Lake, with 58.9% of the total respondents having lived for more than 40 years.

**Table 6:** Resident's status and duration of stay.

Resident's status	No.	%
**Original**	341	66.9
**Migrate**	169	33.1
**Total**	510	100.0
Duration of stay	**No.**	**%**
**20 years and below**	67	13.1
**21 until 40 years**	143	28.0
**41 until 60 years**	186	36.5
**61 years and above**	114	22.4
**Total**	510	100.0

Table 7 shows the results of the analysis of the number of respondent households. A total of 31.8% of respondents have a household of fewer than three people. The number of households between 4 and 6 people is 45.7%. The remaining 22.6% have a household of seven people and above. Detailed analysis showed that the highest number is three people with a percentage of 16.1. Table 8 shows the distribution of the respondents' number of children. According to the distribution of the number of children, 19.8% of respondents did not have children, had five children (13.9%), followed by three people (13.7%) and four people (12.9%).

**Table 7:** Number of households.

Number of Households	No.	%
**None**	6	1.2
**1**	19	3.7
**2**	55	10.8
**3**	82	16.1
**4**	79	15.5
**5**	76	14.9
**6**	78	15.3
**7**	55	10.8
**8**	28	5.5
**9**	20	3.9
**10**	6	1.2
**11**	4	0.8
**12**	1	0.2
**14**	1	0.2
**Total**	510	100.0

**Table 8:** The Number of Household category and number of children.

Category	Number of Households		Number of Children	
	No.	%	No.	%
**None**	6	1.2	101	19.8
**1 until 3 people**	156	30.6	135	26.4
**4 until 6 people**	233	45.7	188	36.8
**7 until 10 people**	109	21.4	75	14.8
**11 people and above**	6	1.2	11	2.2
**Total**	510	100	510	100

Table 9 shows the respondents' education level information, revealing that 7.6% of respondents do not attend school, while up to 8% of respondents have no formal education. According to a detailed analysis based on formal education, 34.9% of respondents had completed primary school, 13.9% had completed lower secondary school, 32.2% had completed upper secondary school, 6.9% had completed STPM/Certificate/Diploma, and 3.7% had a Bachelor's Degree or above.

The article "Assessing wellbeing: Profiling and socioeconomic status of Kenyir Lake side community, Malaysia" was published in 2023. Journal: Heliyon.

**Table 9:** Education level grandfather, father, mother, and respondents.

Education Level	Education Level (Grandfather)		Education Level (Father)		Education Level (Mother)		Education Level (Respondents)	
	No.	%	No.	%	No.	%	No.	%
**Never attend school**	472	92.5	341	66.9	372	72.9	39	7.6
**Primary School**	29	5.7	103	20.2	92	18	178	34.9
**Informal Education**	2	0.4	17	3.3	8	1.6	2	0.4
**Lower Secondary School (SRP/PMR)**	1	0.2	20	3.9	17	3.3	71	13.9
**Upper Secondary School (MCE/SPM)**	4	0.8	21	4.1	17	3.3	164	32.2
**Certificate/STPM/Diploma**	0	0	6	1.2	2	0.4	35	6.9
**Degree and above**	0	0	0	0	0	0	19	3.7
**Other Qualifications (specify)**	2	0.4	2	0.4	2	0.4	2	0.4
**Total**	510	100	510	100	510	100	510	100

The level of education of respondents' mothers and fathers was also studied to further analyse the respondents' level of education (Table 9). It was found that 66.9% and 72.9% of the respondents' fathers and mothers did not attend school. Most respondents' fathers and mothers had education up to primary school with a distribution of 20.2% and 18%, respectively. More specifically, the education level of the grandfather (father's side) was also examined. According to the study's analysis, 92.5% did not attend school. This finding proves that the education level has improved over the years for different generations.

The analysis of this section focuses on the economic variables, namely the employment and income of the respondents. The analysis compares employment types from 10 to 15 years ago to current employment. It also analyses the income from 10 to 15 years ago to the current year's income to comprehend the distribution of current income and past income in detail.

According to Table 10, in the current year, most respondents have basic jobs, which account for 31.4%, followed by self-employment (21.4%), unemployed (15.7%), and people who work in management and service (11.2%). In contrast, the analysis of employment in the last 10–15 years found that 38.2% of respondents were not working, 28% were in basic jobs, 14.5% were self-employed, and 13.3% worked in management and service.

**Table 10:** The differences of main job in the past and current year.

Category	Main Job (10/15 Years before)		Main Job (Current)	
	No.	%	No.	%
**Professional**	16	3.1	24	4.7
**Management and service**	68	13.3	57	11.2
**Business**	14	2.7	50	9.8
**Self-employed**	74	14.5	109	21.4
**Basic job**	143	28	160	31.4
**Retiree**	0	0	30	5.9
**Unemployed**	195	38.2	80	15.7
**Total**	510	100	510	100

Based on the respondent's job category, income distribution was analyzed for the current year and the income of the last 10–15 years. Table 11 shows that 79.2% of the respondents are categorized as poor and extremely poor. A detailed analysis found that 26.3% of respondents had an income below RM580 per month (extremely poor), and 52.9% of respondents had an income between RM581 and RM1500 per month (poor). Only 20.8% of respondents have a monthly income of more than RM1500. Next, an overview of respondents' income over the past 10–15 years revealed that 92% were in the extremely poor category, with 61% having an income below RM580, and 31% having an income around RM581 to RM1500. Only 8% of respondents have a monthly income of more than RM1500.

The article "Assessing wellbeing: Profiling and socioeconomic status of Kenyir Lake side community, Malaysia" was published in 2023. Journal: Heliyon.

**Table 11:** The differences of income in the past and current year.

Income	Main Job (10/15 Years before)		Main Job (Current)	
	No.	%	No.	%
**RM580 and below**	311	61	134	26.3
**RM581 until RM940**	78	15.3	91	17.8
**RM940 until RM1500**	80	15.7	179	35.1
**RM1501 and above**	41	8	106	20.8
**Total**	510	100	510	100

### 4.2 Descriptive analysis (mean) of well-being

According to the Malaysian Family Well-Being Index, family well-being refers to the state of the family being safe, harmonious, and satisfactory. It covers various aspects, namely spiritual, economic and financial, mental, psychosocial, health, political, and sustainability [25].

This study uses a score level of 1–5. According to Ref. [30]; the low, moderate, and high score levels are as shown in Table 12 below.

**Table 12:** Mean score.

Level	Range
Low	1–2.33
Moderate	2.34–3.66
High	3.67–5.00

The average score for the entire Quality of Life/Well-being Index community around Kenyir Lake is 4.08, which is a high level (Table 13). This shows that the community around Kenyir Lake is more satisfied with their quality of life than before.

**Table 13:** Quality of Life/Well-being Index of the community around Kenyir Lake.

No.	Indicator	Very dissatis-fied	Not satisfied	Neutral	Satisfied	Very satisfied	Mean
**1**	Satisfied with current life than before.	1 (0.2)	38 (7.5)	91 (17.8)	202 (39.6)	178 (34.9)	4.02
**2**	Satisfied with current health than before.	0 (0.0)	47 (9.2)	102 (20.0)	204 (40.0)	157 (30.8)	3.92
**3**	Satisfied with achievement in life than before?	1 (0.2)	20 (3.9)	100 (19.6)	220 (43.1)	169 (33.1)	4.05
**4**	Satisfied with current personal relationships with others than before.	1 (0.2)	7 (1.4)	91 (17.8)	238 (46.7)	173 (33.9)	4.13
**5**	Satisfied living as a member of this community than before.	0 (0.0)	13 (2.5)	88 (17.3)	237 (46.5)	172 (33.7)	4.11
**6**	Satisfied with current religious practice than before.	0 (0.0)	7 (1.4)	80 (15.7)	240 (47.1)	183 (35.9)	4.17
**7**	Satisfied with current monthly financial position than before.	2 (0.4)	41 (8.0)	89 (17.5)	229 (44.9)	149 (29.2)	3.95
**8**	Satisfied about recreation with family than before.	0 (0.0)	9 (1.8)	106 (20.8)	233 (45.7)	162 (31.8)	4.07
**9**	Satisfied with current social problems in this place than before.	14 (2.7)	25 (4.9)	118 (23.1)	211 (41.4)	142 (27.8)	3.87
**10**	Satisfied with current safety in this community than before.	0 (0.0)	26 (5.1)	86 (16.9)	240 (47.1)	158 (31.0)	4.04
**11**	Satisfied with current life with family than before.	0 (0.0)	10 (2.0)	73 (14.3)	232 (45.5)	195 (38.2)	4.20
**12**	Satisfied with current engagement with children.	0 (0.0)	2 (0.4)	69 (13.5)	238 (46.7)	201 (39.4)	4.25
**13**	Satisfied about quality time with family.	0 (0.0)	9 (1.8)	74 (14.5)	232 (45.5)	195 (38.2)	4.20
**14**	Balance the work and family?	0 (0.0)	11 (2.2)	81 (15.9)	224 (43.9)	194 (38.0)	4.18
**15**	Satisfied about relationship with partner.	0 (0.0)	5 (1.0)	88 (17.3)	22 0 (43.1)	197 (38.6)	4.19
**16**	Family play their respective roles.	0 (0.0)	13 (2.5)	75 (14.7)	234 (45.9)	188 (36.9)	4.17
**17**	Satisfied with family's problem solving.	0 (0.0)	23 (4.5)	78 (15.3)	232 (45.5)	177 (34.7)	4.10
**18**	Satisfied with family financial management.	2 (0.4)	21 (4.1)	88 (17.3)	214 (42.0)	185 (36.3)	4.10
**19**	Satisfied with family health care.	0 (0.0)	16 (3.1)	76 (14.9)	243 (47.6)	175 (34.3)	4.13
**20**	Satisfied with family safety level.	0 (0.0)	6 (1.2)	70 (13.7)	245 (48.0)	189 (37.1)	4.21
**21**	Satisfied with the role of religion in life.	0 (0.0)	9 (1.8)	70 (13.7)	237 (46.5)	194 (38.0)	4.21
**22**	Satisfied with family's spiritual level.	1 (0.2)	11 (2.2)	71 (13.9)	231 (45.3)	196 (38.4)	4.20
**23**	Satisfied with basic amenities in home.	0 (0.0)	12 (2.4)	75 (14.7)	249 (48.8)	174 (34.1)	4.15
**24**	Satisfied with level of pollution in this place.	2 (0.4)	17 (3.3)	107 (21.0)	231 (45.3)	153 (30.0)	4.01
**25**	Satisfied with family's 3 R practices.	50 (9.8)	77 (15.1)	119 (23.3)	159 (31.2)	105 (20.6)	3.38
**26**	Satisfied with family engagement in term of communication management.	3 (0.6)	14 (2.7)	105 (20.6)	228 (44.7)	160 (31.4)	4.04
**27**	Satisfied with family engagement in communication technology.	0 (0.0)	21 (4.1)	105 (20.6)	233 (45.7)	151 (29.6)	4.01
TOTAL MEAN							**4.08**

The 27 questionnaires above were divided into nine indicators of well-being, namely 1) Life Achievement, 2) Health Level, 3) Family Relationship, 4) Community Relationship, 5) Spiritual Level, 6) Safety Level and Social Problems, 7) Income/Finance, 8) Basic Facilities, and 9) Communication Technology.

The article "Assessing wellbeing: Profiling and socioeconomic status of Kenyir Lake side community, Malaysia" was published in 2023. Journal: Heliyon.

#### 4.2.1 Life achievement indicator

Based on Questions 1 and 3 for Life Achievement indicator, the majority of respondents are satisfied and very satisfied with their lives now compared to before (74.5%) and satisfied and very satisfied with what has been achieved in their lives now compared to before (76.2%). The mean for the life achievement indicator is 4.04 which is at a high level.

#### 4.2.2 Health level indicator

Health aspect is an important thing to be improved in a country to achieve the well-being of the community. Through this study, the majority of respondents (Questions 2, 19, and 26) are satisfied and very satisfied with the health of their lives (70.8%) and their family's health practices (81.9%) compared to before. Most of the respondents are also satisfied with their family's 3 R practices. The mean for the health level indicator is 3.81, which is at a high level.

#### 4.2.3 Family relationship indicator

Family is an important factor in the development of a society. Through this study, the majority (Questions 8, 11, 12, 13, 14, 15, 16, and 17) state that they are satisfied and very satisfied with the time available to do recreational activities with family (77.5%) and satisfied and very satisfied with current life with family than before (83.7%). They also feel satisfied and very satisfied with current engagement with children (86.1%) and having quality time with family (83.7%). Overall, the majority of respondents are satisfied and very satisfied with their relationships with their families. The mean for the family relationship indicator is 4.17 which is at a high level.

#### 4.2.4 Community relationship indicator

The community quality of life approach focuses on the perceptions of community members with what makes life good or not good for them. The relationship with the community is very important in measuring the balance of the quality of life for a person. Through this study, the majority (Questions 4 and 5) state that they are satisfied and very satisfied (80.6%) compared to only 1.6% who are dissatisfied and very dissatisfied with their personal relationships with others now compared to before.

#### 4.2.5 Spiritual level indicator

Spiritual Level is one of the aspects to build self-identity, character, and noble personality among individuals including physical, emotional, spiritual, intellectual, and personality aspects. Based on Table 13, the majority (Questions 6, 21, and 22) of respondents are satisfied and very satisfied with their current religious practice than before (83%) and the role of religion in their life (84.5%). This study also found that only 2.4% of respondents are dissatisfied and very dissatisfied with their family's spiritual practices while 83.7% are satisfied and very satisfied with their family's spiritual practices. The mean for the spiritual level indicator is 4.19 which is at a high level.

The article "Assessing wellbeing: Profiling and socioeconomic status of Kenyir Lake side community, Malaysia" was published in 2023. Journal: Heliyon.

#### 4.2.6 Safety level and social problems indicator

Personal and family safety factors are also important in improving family well-being. From Questions 9, 10, 20, and 24, a total of 78.1% of respondents are satisfied and very satisfied with current social problems in this place than before and 85.1% are satisfied and very satisfied with current safety in this community than before. Next, most respondents are satisfied and very satisfied with the social problems in their place now compared to before (69.2%) and only 7.6% are not satisfied. The majority (75.3%) of them are also satisfied and very satisfied with the level of pollution at their place. The mean for the indicator of safety and social problems is 4.03 which is at a high level.

#### 4.2.7 Income/finance indicator

Income/Finance is a very necessary resource in individual or family life. It allows the individual or family to meet most of the goals and help to stabilise the economic position. It is also a tool to obtain various goods and services that are needed and associated with social status, power, and success. The most important thing is that it is an indicator of the well-being of life. According to Table 13 (Questions 7 and 18), 74.1% of respondents are satisfied and very satisfied with their current monthly financial position than before and the majority of 78.3% are satisfied and very satisfied with their current monthly financial position than before. The mean for the income/financial indicator is 4.03 which is at a high level.

#### 4.2.8 Basic facilities indicator

Infrastructure/Basic facilities can be defined as a physical component of an interconnected system to provide commodities and services needed to enable, maintain, or improve the quality of life of the community [11]. Table 13 (Question 23) shows that the majority of respondents are satisfied with the basic amenities in their homes. The mean for the basic facilities indicator is 4.15 which is at a high level.

#### 4.2.9 Communication technology indicator

The index of well-being also includes modern lifestyle changes based on access to information and communication and technology. Table 13 (Questions 25 and 27) shows that 76.1% of respondents are satisfied and very satisfied with family engagement in terms of communication management and 75.3% of respondents are satisfied and very satisfied with family engagement in communication technology.

The article "Assessing wellbeing: Profiling and socioeconomic status of Kenyir Lake side community, Malaysia" was published in 2023. Journal: Heliyon.

Overall, the average score for the entire Quality of Life/Well-being Index community around Kenyir Lake is 4.08, which is a high level (Table 13). It shows that the community around Kenyir Lake is more satisfied with their quality of life than before.

### 4.3 Descriptive analysis (mean) according to the well-being indicator

Overall, Table 14shows the mean for nine indicators of well-being, namely life achievement, health level, family relationships, community relationships, spiritual level, safety level and social problems, income/finance, basic facilities, and communication technology. Based on Table 14, all indicators have a high mean score. However, the minimum mean value is the health level indicator which is 3.81 and the maximum mean value is the spiritual level indicator which is 4.19.

**Table 14:** Descriptive analysis (mean) according to the well-being indicator.

No.	INDICATOR	MEAN
1.	Life Achievement	4.04
2.	Health Level	3.81
3.	Family Relationships	4.17
4.	Community Relationships	4.12
5.	Spiritual Level	4.19
6.	Safety Level and Social Problems	4.03
7.	Income/Finance	4.03
8.	Basic Facilities	4.15
9.	Communication Technology	4.03

This shows that all the indicator of the respondents are much better than 10 years before. The improvement of their well-being is because of the programmes and activities implemented for them, such as 3 R practices, recreational activities, spiritual programmes (physical, emotional, spiritual, intellectual, and personality aspects), and the development of the infrastructures and facilities.

## 5 Discussion

Overall, according to the data analysis, out of 510 respondents, the majority are male at 77.6%, while female at 22.4%. A total of 89.4% of respondents are aged 36 years and above, while 10.6% are aged 35 years and below. A total of 77.3% of all respondents are married, compared to 22.7% who are divorced, widowed, or single.

The respondents' resident status shows that 66.9% are original residents of Kenyir Lake, with 58.9% of the total respondents have lived for more than 40 years. A number of 86.9% of respondents have lived in Kenyir Lake for more than 20 years, compared to 13.1% of respondents who lived there for less than 20 years.

Based on the respondents’ current job category, the majority have basic jobs at 31.4%, followed by self-employed with a total of 21.4%, 15.7% are unemployed, and 11.2% work in management and service. Generally, 79.2% of the respondents are categorized as poor and extreme poor. A detailed analysis found that 26.3% of respondents have an income below RM580 per month (extremely poor), and 52.9% of respondents have an income between RM581 and RM1500 per month (poor). Only 20.8% of respondents are reported of having a monthly income of more than RM1500.

The article "Assessing wellbeing: Profiling and socioeconomic status of Kenyir Lake side community, Malaysia" was published in 2023. Journal: Heliyon.

Therefore, the findings of this study regarding the respondents' demography profiling indicate that they are still at a poor level. Since the issue of poverty or low income is a multi-dimensional phenomenon beyond a limited reach, it should be viewed as a moral issue that affects humanity itself. Thus, these problems should be taken seriously by several parties, such as the private sector, the government, non-governmental organizations (NGOs), the community, and the individuals themselves.

Nowadays, the main challenge in societal development is to raise living standards in line with rising living costs. The government has provided various development needs that can be enjoyed by all groups to face the challenges of the Industrial Revolution 4.0 (IR4.0). There are nine indicators of well-being in this study, 1) Life Achievement, 2) Health Level, 3) Family Relationship, 4) Community Relationship, 5) Spiritual Level, 6) Safety Level and Social Problems, 7) Income/Finance, 8) Basic Facilities, and 9) Communication Technology. The study shows the average score for the entire Quality of Life/Well-being Index community around Kenyir Lake is 4.08, which is a high level. The findings indicate that the Kenyir Lake Side Community is satisfied with their quality of life.

## 6 Conclusion

Overall, the well-being of the Kenyir Lake side community is high as there are development programmes implemented, especially Kenyir Lake tourism infrastructure, such as water theme parks, Orchid Garden, Kelah Sanctuary, Elephant Sanctuary, Herb Garden, Bird Park, Butterfly Farm, and Duty-free zone, and it indirectly contributes to their economic standard and life satisfaction.

### 6.1 Study limitations

There are several limitations to this study, which could serve as avenues for future research. First, this study limitedly focuses on community at Kenyir Lake only. There could be an in-depth study if the respondents could be from other countries especially in Asia, with various backgrounds of races and religions. The findings too cannot be generalised to other sectors, geographic areas, or industries since other nature and respondents background may not experience the same.

## Compliance with ethical standard

This study has been prepared accordingly and in compliance with ethical standard.

## Funding

We thank 10.13039/501100011891Universiti Malaysia Terengganu for providing funding support for this project (UMT/SRG2018/53275). The authors also thank the Hulu Terengganu District Office for permission to conduct this study.

## Author contribution statement

Norhayati Ab Manaf: Conceived and designed the experiments; Performed the experiments; Analyzed and interpreted the data; Contributed reagents, materials, analysis tools or data; Wrote the paper.

The article "Assessing wellbeing: Profiling and socioeconomic status of Kenyir Lake side community, Malaysia" was published in 2023. Journal: Heliyon.

Nor Hayati Sa'at: Conceived and designed the experiments; Performed the experiments; Wrote the paper.

Nurul Aisyah Awanis A Rahim: Contributed reagents, materials, analysis tools or data.

Siti Nor Adawiyah Azzahra Kamaruddin: Analyzed and interpreted the data.

Siti Salina Abdullah: Conceived and designed the experiments.

Khatijah Omara: Performed the experiments.

## Data availability statement

Data will be made available on request.

## Additional information

No additional information is available for this paper.

## Declaration of competing interest

The authors declare that they have no known competing financial interests or personal relationships that could have appeared to influence the work reported in this paper
